# A Hybrid Multi-Objective Particle Swarm Optimization with Central Control Strategy

**DOI:** 10.1155/2022/1522096

**Published:** 2022-03-09

**Authors:** Meilan Yang, Yanmin Liu, Jie Yang

**Affiliations:** ^1^School of Mathematics and Statistics, Guizhou University, Guiyang 550025, China; ^2^Zunyi Normal University, Zunyi 563002, China

## Abstract

In recent years, researchers have solved the multi-objective optimization problem by making various improvements to the multi-objective particle swarm optimization algorithm. However, we propose a hybrid multi-objective particle swarm optimization (CCHMOPSO) with a central control strategy. In this algorithm, a disturbance strategy based on boundary fluctuations is first used for the updated new particles and nondominant particles. To prevent the population from falling into a local extremum, some particles are disturbed. Then, when the external archive capacity reaches the extreme value, we use a central control strategy to update the external archive, so that the archive solution gets a good distribution. When the dominance of the current particle and the individual best particle cannot be determined, to enhance the diversity of the population, the combination method of the current particle and the individual best particle can be used to update the individual best particle. The experimental results show that CCHMOPSO is better than four multi-objective particle swarm optimization algorithms and four multi-objective evolutionary algorithms. It is a feasible method for solving multi-objective optimization problems.

## 1. Introduction

Multi-objective optimization problems (MOPs) are based on population-based meta-heuristic optimization designs. Generally speaking, MOPs are more challenging than single-objective optimization problems (SOPs). For MOPs [1], there exists a set of optimal solutions to be obtained by a trade-off between different objective values. Meta-inspired optimization algorithms have been widely applied to solve other optimization problems, such as the creation of graphical characters [2], optimal outcomes of evolutionary games [3], and inventory control [4]. Particle swarm optimization (PSO) [5] has been widely used to solve SOPs due to its easy implementation and fast convergence speed. In some research reports [6, 7], the particle swarm optimization algorithm can solve the potential solutions of MOPs very well. Nowadays, in the optimal tuning of fuzzy controller, meta-heuristic slime mould algorithm [8], Takagi-Sugeno type 1 fuzzy logic controller and Takagi-Sugeno type 2 fuzzy logic controller [9] are introduced, which can effectively deal with the fuzzy controller and better solve the optimization problem.

In the research field of MOPs, the purpose was to improve the efficiency of the algorithm and the data structure of the inventory control nondominant vector. Researchers have produced some techniques to maintain the diversity of the population (such as the adaptive grid used by the Pareto archive evolution strategy (PAES) [10]) and the data structure for handling unconstrained external archives (such as dominant tree [11]). To use PSOs for MOPs, at least two issues need to be considered. The first question is how to select learning samples. Since the optimal solution to a MOP is a set, it is difficult to find a solution that performs best on each objective. Since each particle in the population is guided by learning samples to determine the search direction, the selection of learning samples is quite important for PSO, especially for solving MOPs [12]. Therefore, we adopt certain methods to choose the learning samples. The second question is how to balance the convergence and diversity of the population. Because the purpose of multi-objective optimization is to obtain a set of optimal solutions, it is particularly important to maintain the diversity of algorithms. The multi-objective algorithm based on PSO has a fast convergence speed, but it is easy to fall into the local optimum of the MOP. Therefore, the inventory control and algorithmic disturbance strategy are used to maintain the diversity of the population. To address the above problems, researchers have proposed many improved multi-objective particle swarm optimization algorithms (MOPSOs), such as learning samples selected based on Pareto sorting scheme [13], global marginal sorting [14], and learning samples selected based on competition mechanism strategy [15].

In recent ten years, PSO has been widely used in various fields, such as neural network training, industrial production, and hydropower dispatching. When they are used to solve many optimization problems, optimization is to find a solution with the least cost, the best adaptability, and the highest economic benefit among many solutions. For example, Niu et al. proposed a parallel MOPSO [16] to effectively solve the balance between benefit and enterprise output in the operation of cascade hydropower reservoirs. Feng et al. proposed a multi-objective quantum particle swarm optimization [17] to solve the economic environment hydrothermal scheduling optimization problem effectively. Zhang et al. proposed a solution algorithm based on naked particle swarm optimization [18] to effectively solve the problem of reducing the energy consumption of high-energy-consuming buildings. Precup et al. proposed an experiment-based method to teach optimization technology courses in the system engineering curricula at the undergraduate level [19], to solve problems in the optimization, modeling, and control of complex systems.

In this study, we propose a multi-objective particle swarm optimization based on central control and combination methods. CCHMOPSO can deal with MOPs better than PSO algorithms. This algorithm is improved on the MOPSO [20]. In the original algorithm, the update strategy of individual best particles is added, and the perturbation operator is improved. At the same time, the central control strategy was adopted to update the external archive, thus improving the exploratory capacity of particles in the population, while increasing the diversity of the population. These methods help CCHMOPSO to solve MOPs effectively. Compared with some existing MOPSOs, the main contributions of this algorithm are summarized as follows:

1. The study found that during the maintenance of the external archive of MOPSO, 40% of the nondominated solutions are randomly deleted from the grid with the highest density in the archive. This method will blindly delete good nondominated solutions, and it will affect the search results of particles. Therefore, this study designs a new central control method, which deletes the nondominated solution according to the distribution of the solution and the Euclidean distance from the central particle. It can improve the quality of the solution in the archive and accelerate the convergence speed of the algorithm. This helps guide the search direction of the particles towards the true Pareto front.
2. For the traditional MOPSO, the individual optimal particle is selected by comparing the value of the objective function. When the objective function value between two particles cannot be compared, it is selected randomly. If the individual optimal particle is selected improperly, it is easy to be trapped in local optimization. Therefore, the algorithm introduces a combination method to update the individual optimal location, which can enhance the diversity of the population and avoid falling into local optimization. This helps guide the particles to search for the globally optimal particles.
3. In CCHMOPSO, nondominant particles and new particles are obtained after each update implements an improved mutation strategy. This method effectively prevents particles from falling into local optima, so that nondominant particles have a chance to become dominant. However, perturbing the particles can help the particles to search for the global optimal particle.

The advantages of CCHMOPSO are verified by experiments. In the experiment, 22 standard test problems are used for verification and compared with four improved MOPSOs and four extremely competitive MOEAs: CMOPSO [15], MOPSOCD [21], MPSOD [12], NMPSO [22], MOEAD [23], NSGA-II [24], SPEA2 [25], and MOEAIGDNS [26]. The experimental results show that CCHMOPSO's overall performance is better than other eight algorithms in terms of solution set quality.

The specific work of the study is as follows. The second section reviews the MOP, briefly introduces the PSO, and the existing MOPSO. The third section gives the details of CCHMOPSO proposed in this study. The fourth section is the research comparison and relevant discussion. The fifth section summarizes this study.

## 2. Related Work

### 2.1. Multi-Objective Optimization

Many optimization problems in the engineering field require simultaneous optimization of multiple different objectives. This kind of problem is called MOP, in which the objectives to be optimized often conflict with each other. Therefore, the multi-objective optimization algorithm is mainly to find a set of relatively optimal solutions between various objectives in the solution space, and the more uniform the distribution of these solutions, the better. In general, the multi-objective optimization problem (taking the minimization problem as an example) is expressed as follows:

(1) $$\begin{array}{c} \text{Min}\overset{⟶}{F}\left(\overset{⟶}{x}\right)=\left(f_{1}\left(\overset{⟶}{x}\right),f_{2}\left(\overset{⟶}{x}\right),...,f_{M}\left(\overset{⟶}{x}\right)\right),\\ \overset{⟶}{x}=\left(x_{1},x_{2},...,x_{D}\right)\in \Omega \subset R^{D}. \end{array}$$

where $\overset{⟶}{x}=\left(x_{1},x_{2},...,x_{D}\right)$ is represented as a *D*-dimensional vector of independent variables; *f*_*i*_ : Ω⟶*R*(*i*=1,2, ..., *M*), *M* is the dimension of the target space, and $\overset{⟶}{F}\left(\overset{⟶}{x}\right)$ is the minimization of *M* objects. The following are some related concepts in the multi-objective optimization problem.

**Definition 1 .**

(Pareto domination): let $\overset{⟶}{x}$ and $\overset{⟶}{y}$ be two solutions of multi-objective optimization problem (1). If

(2) $$\begin{array}{c} \forall i=1,2,...,M:f_{i}\left(\overset{⟶}{x}\right)\leq f_{i}\left(\overset{⟶}{y}\right)\wedge \exists j\in 1,2,...,M:f_{j}\left(\overset{⟶}{x}\right)<f_{j}\left(\overset{⟶}{y}\right). \end{array}$$

then it is said that $\overset{⟶}{x}$ dominates $\overset{⟶}{y}$, denoted as $\overset{⟶}{x}≺\overset{⟶}{y}$.

**Definition 2 .**

(Pareto optimal solution): let $\overset{⟶}{x}$ be the solution of the multi-objective optimization problem (1). If

(3) $$\begin{array}{c} ￢\exists \overset{⟶}{y}\in \Omega :\overset{⟶}{y}≺\overset{⟶}{x}. \end{array}$$

then $\overset{⟶}{x}$ is called the Pareto optimal solution or nondominated solution.

**Definition 3 .**

(Pareto optimal solution set): the set of all Pareto optimal solutions in the decision space $\overset{⟶}{x}$ is called the Pareto optimal solution set (Pareto optimal set, PS), i.e.,

(4) $$\begin{array}{c} PS=\left\{\overset{⟶}{x}|￢\exists \overset{⟶}{y}\in \Omega :\overset{⟶}{y}≺\overset{⟶}{x}\right\}. \end{array}$$

**Definition 4 .**

(Pareto front): in the Pareto optimal solution set, the curve (surface) formed by the objective space is called Pareto front, i.e.,

(5) $$\begin{array}{c} PF=\left\{\overset{⟶}{F}\left(\overset{⟶}{x}\right)=\left(f_{1}\left(\overset{⟶}{x}\right),f_{2}\left(\overset{⟶}{x}\right),...,f_{M}\left(\overset{⟶}{x}\right)\right)|\overset{⟶}{x}\in PS\right\}. \end{array}$$

Figure 1 plots the Pareto front of a special case of a bi-objective optimization function.

### 2.2. Particle Swarm Optimization

The particle swarm optimization (PSO) was originally developed by Kennedy and Eberhart [5] for optimization problems. The PSO was inspired by the foraging behavior of bird flocks. In PSO, individuals are flying in a multidimensional space in groups, to find the potential optimal solution in the population. It is worth noting that each individual learns from their past individual experience and the experience of successful peers and updates their speed and position adaptively. In the standard PSO [27], the individuals in the swarm are called particles, and it is a potential solution in the swarm. The position and velocity of the particles are updated according to the following formula:

(6) $$\begin{array}{c} v_{ij}\left(t+1\right)=wv_{ij}\left(t\right)+c_{1}r_{1}\left(x_{p{\text{best}}_{ij}}\left(t\right)-x_{ij}\left(t\right)\right)+c_{2}r_{2}\left(x_{g{\text{best}}_{j}}\left(t\right)-x_{ij}\left(t\right)\right), \end{array}$$

(7) $$\begin{array}{c} x_{ij}\left(t+1\right)=x_{ij}\left(t\right)+v_{ij}\left(t+1\right). \end{array}$$

where $\overset{⟶}{x_{i}}=\left(x_{i1},x_{i2},...,x_{i\;D}\right)$ and $\overset{⟶}{v_{i}}=\left(v_{i1},v_{i2},...,v_{i\;D}\right)$ represent position and velocity of the *i*th particle in the *D*th dimensional search space; *x*_*p*best_*ij*__ represents the individual optimal *j*th dimensional position of the *i*th particle and is usually called the individual optimal position (pbest); *x*_*g*best_*j*__ represents the *j*th dimensional position of the globally optimal particle in the population and is usually called the global optimal position (gbest); *w* is the coefficient of inertia, *w* = 0.4; *c*_1_ and *c*_2_ represent the acceleration coefficients, *c*_1_=*c*_2_=2.0; *r*_1_ and *r*_2_, respectively, represent two random coefficients generated uniformly in the range of [0, 1]; and *t* represents the number of iterations, *t*=1,2, ..., *T* (*T* is the maximum number of iterations). In general, to keep the particles from flying out of the search space, a maximum value (*v*_max_) is defined for each dimension of the particle's velocity vector. When the particle velocity *v*_*ij*_ exceeds the defined *v*_max_, the particle velocity *v*_*ij*_ is directly set to *v*_max_.

### 2.3. Existing Multi-Objective Particle Swarm Optimization Algorithms

In recent years, some MOPSOs have been proposed. Next, we briefly review some representative MOPSOs.

The algorithm was proposed by Coello et al. [6], which used the Pareto dominance relationship to determine the learning samples, and stored the nondominated particles in an external archive. Although the MOPSO performed better than the traditional MOEAs in solving MOPs, such as NSGA-II [24] and PAES [10], it was difficult to solve MOPs in complex landscape. Aiming at the problem that the learning samples in the MOPSO are determined by the dominance relationship, Zhang et al. [23] were based on the decomposition-based MOPSO and replaced the genetic operator with a search method based on the PSO algorithm. Dai et al. [12] proposed another decomposition method of MOPSO, which divided the target space vector into subregions based on a set of direction vectors.

In the MOPSO, some methods to enhance the diversity of the population have been proposed. Zhang et al. [15] proposed a MOPSO based on a competition mechanism, in which a competition mechanism was used to select the global optimal solution. Liu et al. [22] proposed a MOPSO that balances fitness estimation methods, in which the algorithm adopted a new update formula to enhance the convergence of the algorithm. Lin et al. [28] proposed a MOPSO where the PSO-based search method searched for particles in the population with crossover [24] and mutation operation [29] updated the particles in the archive. Gu et al. [30] proposed MOPSO based on R2 contribution and adaptive method, in which a new global optimal solution selection mechanism was adopted to maintain the diversity of the population. These algorithms could avoid falling into local optima and enhanced the diversity of the population.

In recent years, researchers have proposed some hybrid swarm intelligence algorithms. For example, Liu et al. proposed a particle swarm optimizer [31] that simulates human social interaction behavior. The learning strategy of this algorithm makes full use of the excellent information of each particle to guide the particle search, which improves the diversity of the population. Liu et al. proposed a PSO based on genetic interference hybrid learning [32], which uses the genetic interference hybrid strategy to update particles and improves the ability of the population to avoid falling into local optimal solutions. Qian et al. proposed an improved genetic algorithm [33] based on memory update and environmental response scheme, which uses memory update and environmental response scheme to improve the adaptability of the algorithm to different dynamic environments. Leng et al. proposed MOPSO based on optimal grid distance [34], which integrates two grid sorting methods in maintaining the size of the external archives. Niu et al. proposed a bacterial foraging optimization algorithm [35] based on a coevolutionary structure redesign, so that all bacteria can learn from each other and search for the optimal solution cooperatively, which can speed up convergence and promote search accuracy. Moattari et al. discussed a brain-inspired approach to design evolutionary optimization algorithm [36]. Kaur et al. designed silicon fin-shaped field-effect transistor devices on insulators and the best indicators. After using a set of parameters to train the neural network and determine the fitness function, they realized the genetic algorithm and the whale optimization algorithm [37].

In summary, the main concern of the existing MOPSO is how to effectively improve the diversity of the population. In this study, a MOPSO based on central control and combination method (CCHMOPSO) is proposed. In CCHMOPSO, a new strategy is proposed to improve the MOPSO. This central control method combines the Euclidean distance to maintain the external archive size that can improve the quality of the solution. In addition, a new method is proposed to update the best position of individuals, which enhances the diversity of the population in a combined manner. The details of the algorithm will be introduced in Section 3.

## 3. Description of CCHMOPSO Algorithm

In this section, we first elaborate on three improvement strategies of the CCHMOPSO and then give the basic framework of the CCHMOPSO.

### 3.1. Central Control Strategy for External Archiving

The purpose of external archiving is to preserve the high-quality nondominated solutions found during the search process. In the early stage of the algorithm, there are few nondominant solutions, so archiving can effectively preserve the dominant nondominant solutions. In the late stage of the algorithm, since the population has a limited search range in the feasible domain space, it is necessary to consider whether the capacity of the archive is full. Therefore, we need to maintain the external archive to guide the population to search to the Pareto front and ensure the distribution of solutions on the Pareto front. When the number of nondominated solutions generated by the algorithm exceeds the maximum capacity of the archive, some particles need to be deleted from the archive. This study proposes a central control strategy in the external archive to update the archive. This strategy deletes some particles one by one from the archive, while storing high-quality nondominated solutions. Next, we will describe the update of the external store in detail.

During each iteration of PSO, it generates a set of nondominated solutions (where this set of nondominated solutions is the relatively dominant solutions obtained by the Pareto nondominated ranking [38], and no solution among them is superior to several other solutions). Compared with this set of nondominated solutions with the individuals in the external repository one by one (where the external repository is initially empty), the method of selecting the dominant particle or two nondominant particles obtained after each comparison can be described as follows: (1) both dominant and nondominant solutions are stored in the external archive, while the dominant and nondominant solutions in the archive are retained; (2) when the capacity of the external archive is within the size limit, all dominant and mutually exclusive nondominant solutions are stored in the external archive; and (3) when the capacity reaches the limit, this study uses a central control strategy to delete some particles one by one and at the same time store the dominant nondominated solutions one by one.

When the capacity of the external archive reaches its limit, an adaptive grid [10] is first established, and then, a method to delete some particles in the archive is used. In the original MOPSO [20], objects were removed based on the density of the grid. It was based on the idea that the greater the density of the grid, the greater the probability that particles within it would be deleted. It randomly deleted some particles from the grid with the highest density according to a certain proportion. Although this method guarantees the scale of the archive, it has a certain degree of blindness and will bring difficulties to the population to converge. Therefore, the update and maintenance strategy of the external archive are very critical for the MOPSO. In this study, a central control strategy is used to determine the object to be deleted. The determinant factor depends on the grid density and the Euclidean distance from the central particle. The basic idea is to use the adaptive grid in the external storage and find the central particle from the densest grid of the adaptive grid and mark it as *N*^*∗*^. To get a good distribution, we select 40% [20] of the total number of particles from the densest grid and delete it. (8) calculates the total number *q* of deleted particles in the densest grid; (9) and (10), respectively, calculate the distances *d*_*i*_^*∗*^ and *d*_*i*_ between the central particle *N*^*∗*^ and the *i*th individual on the left and right sides. We need to delete the *q* particles with the smallest distance in front of them in sequence, and the specific method is as follows: (1) if the total particle number in the densest grid is an odd number, the middle particle in the grid is directly selected as the central particle *N*^*∗*^, and the *q* particles with the smallest distance in front are deleted one by one (Figure 2(a)); (2) if the total particle number in the densest grid is even, one of the two particles in the middle of the grid is randomly selected as the central particle *N*^*∗*^, and then, the *q* particles with the smallest distance in front are deleted one by one (Figures 2(b) and 2(c)). It is worth noting that deleting particles one by one in the archive also stores the dominant nondominated solutions one by one.

(8) $$\begin{array}{c} q=\left[s\cdot 0.4\right], \end{array}$$

(9) $$\begin{array}{c} d_{i}^{*}={|\overset{⟶}{x}}_{N^{*}}-{\overset{⟶}{x}}_{N^{*}-i}|, \end{array}$$

(10) $$\begin{array}{c} d_{i}={|\overset{⟶}{x}}_{N^{*}}-{\overset{⟶}{x}}_{N^{*}+i}|, \end{array}$$

where represents the rounding conforms; *| |* represents Euclidean distance; *s* represents the total number of individuals in the densest cell; ${\overset{⟶}{x}}_{N^{*}}$ represents the position of the central particle; ${\overset{⟶}{x}}_{N^{*}-i}$ represents the *i*th individual position to the left of the central particle; and ${\overset{⟶}{x}}_{N^{*}+i}$ represents the *i*th individual position to the right of the central particle.

When the external archive is updated each time, some particles closest to the central particle in the most densely distributed area of the archive are deleted according to the central control strategy. It can maintain the diversity of the solution set and ensure that the solutions in the external archive have a good distribution.

### 3.2. Update Strategy of Individual Optimal Particle

In PSO, the individual best position (*pbest*) of a particle is the best position obtained by itself so far. Reasonable selection of *pbest* is conducive to enhancing the population's ability to develop local space, so that particles can find the optimal solution in multiple regions. When solving SOPs, we only need to compare whether the fitness value of the current particle is better than the fitness value of the *pbest* to determine the *pbest*. However, in the MOPs, the best individual is chosen by the information of the externally archived solution. In this study, the individual best particle update strategy is adopted, and the Pareto dominance relationship is used to update the individual best particle, so as to improve the convergence speed. After the individual best particles are updated, it is also necessary to maintain the particles in the feasible region space to prevent them from exceeding the boundary of the space (avoid newly generated particles not in the effective feasible region space).

The dominance relationship between the current particle and best individual is first compared. There are three situations as follows: (1) if the individual best particle dominates the current particle, the individual best particle remains unchanged; (2) otherwise, the current particle dominates the individual best particle, and the current particle replaces the individual best particle; and (3) if they do not dominate each other, it is difficult to choose a single one as the individual best solution. Therefore, the text uses a combined method [39] to update the individual best particles, which is conducive to the search of the population particles in their own local space and improves the development ability of the algorithm. At the same time, it also enhances the diversity of the population and avoids the ability to fall into local minima. The updated formula of the best individual is as follows:

(11) $$\begin{array}{c} {\overset{⟶}{x}}_{p{\text{best}}_{i}}\left(t+1\right)=\left\{\begin{array}{cc} {\overset{⟶}{x}}_{i}\left(t+1\right), & f\left({\overset{⟶}{x}}_{p{\text{best}}_{i}}\left(t\right)>f\left({\overset{⟶}{x}}_{i}\left(t+1\right)\right)\right),\\ {\overset{⟶}{x}}_{p{\text{best}}_{i}}\left(t\right), & f\left({\overset{⟶}{x}}_{p{\text{best}}_{i}}\left(t\right)<f\left(\left({\overset{⟶}{x}}_{i}\left(t+1\right)\right)\right.\right),\\ u{\overset{⟶}{x}}_{i}\left(t+1\right)+c\left(1-u\right){\overset{⟶}{x}}_{p{\text{best}}_{i}}\left(t\right), & f\left({\overset{⟶}{x}}_{p{\text{best}}_{i}}\left(t\right)\right)=f\left({\overset{⟶}{x}}_{i}\left(t+1\right)\right), \end{array}\right. \end{array}$$

where parameter *u* represents the uniform factor, the function of this factor is to balance the influence of the search directions of the two solutions: if *u* = 1, the position of the current particle is selected as *pbest*, ${\overset{⟶}{x}}_{pbest_{i}}\left(t+1\right)={\overset{⟶}{x}}_{i}\left(t+1\right)$; if *u* = 0, the *pbest*, ${\overset{⟶}{x}}_{p{\text{best}}_{i}}\left(t+1\right)={\overset{⟶}{x}}_{p{\text{best}}_{i}}\left(t\right)$, is kept. On the other hand, parameter *u* (*u* ∈ [0, 1]) is the compound searchability of two solutions, which combines the respective advantages of the two solutions, *u* = 0.1; *c* ~ *N*(0, 0.01^2^*I*) is normally distributed parameters, and *I*_*D*×*D*_ is the identity matrix; parameter *c* is a random parameter that mimics the mutation of the evolutionary algorithm to enhance the exploration ability of the algorithm.

A dual-objective optimization problem is taken as an example: assuming that the objective function value of the current particle *i* in the *t* + 1 th iteration is $f\left({\overset{⟶}{x}}_{i}\left(t+1\right)\right)=\left(f_{1}\left({\overset{⟶}{x}}_{i}\left(t+1\right)\right),f_{2}\left({\overset{⟶}{x}}_{i}\left(t+1\right)\right)\right)$, the objective function value of the best individual is $f\left({\overset{⟶}{x}}_{p{\text{best}}_{i}}\left(t\right)\right)=\left.\left(f_{1}\left({\overset{⟶}{x}}_{p{\text{best}}_{i}}\left(t\right)\right.\right),f_{2}\left({\overset{⟶}{x}}_{p{\text{best}}_{i}}\left(t\right)\right)\right)$. In this study, the individual best particle update strategy for particles is as follows:

(12) $$\begin{array}{c} \left(1\right)\left.\begin{array}{c} f_{1}\left({\overset{⟶}{x}}_{i}\left(t+1\right)\right)<f_{1}\left({\overset{⟶}{x}}_{p{\text{best}}_{i}}\left(t\right)\right),f_{2}\left({\overset{⟶}{x}}_{i}\left(t+1\right)\right)<f_{2}\left({\overset{⟶}{x}}_{p{\text{best}}_{i}}\left(t\right)\right)\\ f_{1}\left({\overset{⟶}{x}}_{i}\left(t+1\right)\right)<f_{1}\left({\overset{⟶}{x}}_{p{\text{best}}_{i}}\left(t\right)\right),f_{2}\left({\overset{⟶}{x}}_{i}\left(t+1\right)\right)=f_{2}\left({\overset{⟶}{x}}_{p{\text{best}}_{i}}\left(t\right)\right)\\ f_{1}\left({\overset{⟶}{x}}_{i}\left(t+1\right)\right)=f_{1}\left({\overset{⟶}{x}}_{p{\text{best}}_{i}}\left(t\right)\right),f_{2}\left({\overset{⟶}{x}}_{i}\left(t+1\right)\right)<f_{2}\left({\overset{⟶}{x}}_{p{\text{best}}_{i}}\left(t\right)\right) \end{array}\right\}{\overset{⟶}{x}}_{p{\text{best}}_{i}}\left(t+1\right)={\overset{⟶}{x}}_{i}\left(t+1\right),\\ \left(2\right)\left.\begin{array}{c} f_{1}\left({\overset{⟶}{x}}_{i}\left(t+1\right)\right)>f_{1}\left({\overset{⟶}{x}}_{p{\text{best}}_{i}}\left(t\right)\right),f_{2}\left({\overset{⟶}{x}}_{i}\left(t+1\right)\right)>f_{2}\left({\overset{⟶}{x}}_{p{\text{best}}_{i}}\left(t\right)\right)\\ f_{1}\left({\overset{⟶}{x}}_{i}\left(t+1\right)\right)>f_{1}\left({\overset{⟶}{x}}_{p{\text{best}}_{i}}\left(t\right)\right),f_{2}\left({\overset{⟶}{x}}_{i}\left(t+1\right)\right)=f_{2}\left({\overset{⟶}{x}}_{p{\text{best}}_{i}}\left(t\right)\right)\\ f_{1}\left({\overset{⟶}{x}}_{i}\left(t+1\right)\right)=f_{1}\left({\overset{⟶}{x}}_{p{\text{best}}_{i}}\left(t\right)\right),f_{2}\left({\overset{⟶}{x}}_{i}\left(t+1\right)\right)>f_{2}\left({\overset{⟶}{x}}_{p{\text{best}}_{i}}\left(t\right)\right) \end{array}\right\}{\overset{⟶}{x}}_{p{\text{best}}_{i}}\left(t+1\right)={\overset{⟶}{x}}_{p{\text{best}}_{i}}\left(t\right),\\ \left(3\right)\left.\begin{array}{c} f_{1}\left({\overset{⟶}{x}}_{i}\left(t+1\right)\right)>f_{1}\left({\overset{⟶}{x}}_{p{\text{best}}_{i}}\left(t\right)\right),f_{2}\left({\overset{⟶}{x}}_{i}\left(t+1\right)\right)<f_{2}\left({\overset{⟶}{x}}_{p{\text{best}}_{i}}\left(t\right)\right)\\ f_{1}\left({\overset{⟶}{x}}_{i}\left(t+1\right)\right)<f_{1}\left({\overset{⟶}{x}}_{p{\text{best}}_{i}}\left(t\right)\right),f_{2}\left({\overset{⟶}{x}}_{i}\left(t+1\right)\right)>f_{2}\left({\overset{⟶}{x}}_{p{\text{best}}_{i}}\left(t\right)\right)\\ f_{1}\left({\overset{⟶}{x}}_{i}\left(t+1\right)\right)=f_{1}\left({\overset{⟶}{x}}_{p{\text{best}}_{i}}\left(t\right)\right),f_{2}\left({\overset{⟶}{x}}_{i}\left(t+1\right)\right)=f_{2}\left({\overset{⟶}{x}}_{p{\text{best}}_{i}}\left(t\right)\right) \end{array}\right\}{\overset{⟶}{x}}_{p{\text{best}}_{i}}\left(t+1\right)={\overset{⟶\prime }{x}}_{p{\text{best}}_{i}}\left(t+1\right),\\ {\overset{⟶\prime }{x}}_{p{\text{best}}_{i}}\left(t+1\right)=u{\overset{⟶}{x}}_{i}\left(t+1\right)+c\left(1-u\right){\overset{⟶}{x}}_{p{\text{best}}_{i}}\left(t\right). \end{array}$$

### 3.3. Perturbation Strategy Based on Boundary Fluctuation

The implementation of perturbation strategy in PSO (e.g., RPSO [40]) can promote the searchability of particles, because perturbation strategy helps to enhance the diversity of population and make particles get rid of local optimization. The following situations may occur in the population. When a particle is searching in the feasible region space, if the particle finds a good position, then other particles will fly in its direction. It should be noted that if the good position explored by the particle corresponds to the local optimal solution, then our particle cannot search the entire feasible region space. As a result, the diversity of the population will be lost and the algorithm will fall into a local optimum [41, 42]. To avoid the above situation and enhance the diversity of solutions, this study introduces a perturbation strategy to improve the diversity of search solutions in the process of CCHMOPSO optimization. The disturbed objects are the nondominant particles and the new particles after the update. This strategy is affected by the exponential coefficient to randomly select particles, which are first perturbed with convergent upper bounds. If the result of the perturbation causes the particle position to exceed the upper bound, then the perturbation towards the lower bound will be carried out. This is beneficial to reduce the probability of the algorithm falling into a local optimum and maintain the diversity of the population. From the calculation of (13), it can be seen that the perturbation amplitude of the particles will decrease with the increase in the number of iterations. In the perturbation operation, the disturbed range of the whole population gradually decreases, and the algorithm converges as the disturbed particles gradually decrease. The perturbation formula is as follows:

(13) $$\begin{array}{c} \psi =\exp\left(\frac{-5t}{T}\right), \end{array}$$

(14) $$\begin{array}{c} x_{ij}=x_{ij}+\psi ,i=1,2,...,n,j=j^{*}\left(i\right),j^{*}=\text{fix}\left(\text{rand}\left(n\;D\right)+1\right), \end{array}$$

(15) $$\begin{array}{c} x_{ij}=\left\{\begin{array}{cc} x_{ij}, & x_{ij}\leq ub_{i},\\ ub_{i}-r_{3}\psi , & x_{ij}>ub_{i}, \end{array}\right. \end{array}$$

where $\overset{⟶}{ub}$ represents the upper bound of particle position, $\overset{⟶}{ub}=\left(1,1,...,1\right)$; *ψ* is an exponential disturbance factor, which will decrease as the number of *t* iterations increases, the *ψ* coefficient decreases, and the disturbance range decreases; *n* (*n* *≤* *N*) represents the number of particles affected by the perturbation factor; *j* (*j* *≤* *D*) represents the specific position of *i*th particle disturbance, which is affected by the number of iterations; *r*_3_ represents the random coefficient uniformly distributed within the range of [0, 1]; and *T* represents the maximum number of iterations.

New particles obtained after each update, and all nondominant particles after each external archive update, adopt a perturbation strategy for these particles. Using perturbation, the diversity of solutions is enhanced, and some particles become feasible, which effectively avoids the population falling into local extremum.

All in all, the abovementioned perturbation strategy makes the particles converge to the true Pareto front faster and accelerates the convergence speed. It is worth noting that compared with the traditional MOPSO, CCHMOPSO proposed in the text does not increase the amount of calculation too much.

### 3.4. Framework of CCHMOPSO

The description of CCHMOPSO is as follows:

  Step 1. Initialization. First, set relevant parameters, such as population size *N* and final stop condition *T*_max_=10000. Secondly, set the archive to an empty set, and set the initial velocity $\overset{⟶}{v}=0$ and position $\overset{⟶}{x}$ of the initialized particles;
  Step 2. Perturb the particles in the population using the methods described in Section 3.3;
  Step 3. Calculate the objective function value of all particles in the population;
  Step 4. Update the external archive using the methods shown in Section 3.1;
  Step 5. Update the position of pbest and gbest (use (11) in Section 3.2 to update the position of pbest);
  Step 6. Update the velocity and position using (6) and (7);
  Step 7. Use the method described in Section 3.3 to perform disturbing effects on new particles in the population;
  Step 8. Calculate the objective function value of all new particles in the population;
  Step 9. Update the external archive again using the methods described in Section 3.1;
  Step 10. Use the method described in Section 3.3 again to perform disturbing effects on nondominant particles;
  Step 11. Update the position of pbest and gbest (use (11) in Section 3.2 to update the position of pbest);
  Step 12. Judge whether the algorithm reaches the final stop condition. If yes, stop and output the final result; otherwise, return to step 6.

Figure 3 shows a flowchart of CCHMOPSO.

## 4. Validation Results

In this section, several experiments are performed to verify the performance of CCHMOPSO. The content of this section is divided into four parts for description. The first part is the performance index; the second part is parameter setting; the third part is the comparison between CCHMOPSO and four other MOPSOs; and the fourth part compares CCHMOPSO with four competitive MOEAs.

### 4.1. Performance Indicators

In this study, two performance metrics are used to compare CCHMOPSO with selected MOPSOs and MOEAs. These metrics are the inverted generational distance and hyper-volume.

The inverted generational distance [43] (IGD) metric is used to evaluate the performance of the nine algorithms. Normally, this indicator is used to measure the distance between the true Pareto front and the nondominated solution set obtained by the algorithm. The IGD value is a metric, and its function is to evaluate the quality of the solution set obtained in terms of convergence and diversity. The smaller the IGD value, the better the quality of the solution set obtained by the algorithm. In addition to evaluating the performance of the algorithm, it is also necessary to further evaluate the overall performance of the algorithm. IGD is defined as follows:

(16) $$\begin{array}{c} \text{IGD}\left(P\right)=\frac{\sum_{i=1}^{\left|F^{*}\right|}\text{dist}\left(x_{i}^{*},P\right)}{\left|F^{*}\right|}, \end{array}$$

where *P* represents the current Pareto front set; dist(*x*^*∗*^, *P*) represents the Euclidean distance between a point *x*^*∗*^ ∈ *F*^*∗*^ and the nearest solution in *P*.

The hyper-volume [44] (HV) metric is used to evaluate the overall performance of the nine algorithms. This metrics is achieved by measuring the hyper-volume of the region composed of the optimal set and the reference point in the target space. Its function is to evaluate the distribution and convergence. The larger the HV value, the better the overall performance obtained by the algorithm. The reference point of HV is set to (1.1, 1.1).

(17) $$\begin{array}{c} HV\left(P\right)=\text{Leb}\left(\underset{x\in P}{\cup }\left[f_{1}\left(\overset{⟶}{x}\right),R_{1}\right]\times \cdots \times \left[f_{M}\left(\overset{⟶}{x}\right),R_{M}\right]\right), \end{array}$$

where *f*_*i*_ represents the *i*th objective function value of *P*; *R*_*i*_ represents the *i*th objective function value of the reference point. HV value is set as (1.1, 1.1).

### 4.2. Parameter Setting

To verify the effectiveness of the proposed algorithm, four typical MOPSOs are selected for performance comparison, namely CMOPSO [15], MOPSOCD [21], MPSOD [12], and NMPSO [22]; four competitive MOEAs are also selected for performance comparison, namely MOEAIGDNS [26], SPEA2 [25], NSGA-II [24], and MOEAD [23]. We use 22 benchmark problems in the three test series of ZDT [45], DTLZ [46], and UF [47] to evaluate the performance of nine algorithms, of which ZDT1 to ZDT4 and ZDT6, and UF1 to UF7 are all dual goal test problem; DTLZ1 to DTLZ7 and UF8 to UF10 are all three-objective test problems. For the dual-objective test problem, the number of decision variables in ZDT1 to ZDT3 and UF1 to UF7 is set to 30, and the number of decision variables in ZDT4 and ZDT6 is set to 10. For the three-objective test problem, the number of decision variables in DTLZ1, DTLZ7, DTLZ2 to DTLZ6, and UF8 to UF10 is set to 7, 22, 12, and 30, respectively. These parameters are customized for the test problem.

To make a fair comparison, the relevant parameters of all the comparison algorithms used in this study are set according to the recommended values in Table 1. *p*_*c*_ and *p*_*m*_ represent the crossover and mutation probability, respectively; *η*_*c*_ and *η*_*m*_ represent the distribution indicators, respectively. For CMOPSO and MOPSOCD, their control parameter *R* is randomly sampled in [0, 1], and the inertia weight *w* of MOPSOCD is 0.4; for MPSOD and CCHMOPSO, their control parameter *c* is 2.0, and the inertia weight *w* of MPSOD is randomly sampled in [0.1, 0.9], while the inertia weight *w* of CCHMOPSO is 0.4. For NMPSO, the control parameter *c* is randomly in [1.5, 2.5]. For MOEAD, *T* represents the neighborhood size between weight coefficients, and *F* represents the crossover probability of differential evolution. The div of CCHMOPSO represents the number of division grids of cells. In this study, the population size of all algorithms is set to *N* = 200. Except that the maximum number of fitness assessments for test problem ZDT4 is 40000, the maximum number of fitness assessments for other 21 test problems is 10000. On each test question, the experiment is carried out with 30 independent runs, and each result of IGD value and HV value and their average and standard deviation were recorded. In this article, all the algorithm source codes used for comparison are provided in PlatEMO [48].

### 4.3. Comparison Experiments with Four MOEAs

As shown in Tables 2 and 3, the mean and standard deviation of the IGD value and HV value of the five algorithms on 22 test problems are given. The five algorithms are as follows: MOEAIGDNS, SPEA2, NSGA-II, MOEAD, and CCHMOPSO algorithms. Then, the best IGD and HV values of the five algorithms in 22 test problems are recorded, and the IGD and HV values of the corresponding algorithms are marked in bold.

Tables 2 and 3 show the result comparison of the index IGD value and HV value obtained among the five algorithms. Compared with existing MOEAs, CCHMOPSO has achieved better overall performance on test problems. It can be seen from the IGD value that among the 22 test problems, the CCHMOPSO, NSGA-II, MOEAIGDNS, SPEA2, and MOEAD algorithms obtain the best average performance on 13, 5, 1, 2, and 1 test problems, respectively. Therefore, in the 22 test problems, the IGD value obtained by CCHMOPSO is better than the other four algorithms. It is found from Table 2 that CHHMOPSO significantly outperforms the other four algorithms on the test problems UF1-UF7. Because it uses a central control method to maintain external archives and improve the search capabilities of the algorithm, in the 22 comparisons, the effect of CCHMOPSO is better than that of MOEAIGDNS, SPEA2, NSGA-II, and MOEAD for 16, 14, 13, and 17 times, respectively. However, it is only 6, 8, 9, and 5 times worse than MOEAIGDNS, SPEA2, NSGA-II, and MOEAD, respectively. For the test problems, DTLZ5 and DTLZ6 of degraded PFs, MOEAD, SPEA2, and MOEAIGDNS perform poorly because they use evolutionary search and cannot effectively solve the test problems DTLZ5 and DTLZ6. Therefore, in terms of index IGD, CCHMOPSO has the better performance compared with the other four algorithms in most of the 22 test problems.

To further verify the effectiveness of CCHMOPSO, an important test index HV is used in addition to the index IGD value. As can be seen from the HV values, CCHMOPSO, NSGA-II, MOEAD, MOEAIGDNS, and SPEA2 obtain the best overall performance on 15, 3, 1, 1, and 1 of the 22 test problems, respectively. Therefore, the CCHMOPSO obtains relatively better HV values than the other four algorithms in the 22 test problems. Note that in test problems ZDT3 and DTLZ7, the IGD values obtained by our CCHMOPSO are relatively average, but it can be seen from the HV values that it has the best overall performance.

As shown in Figure 4, the box plot of IGD index results of five algorithms is drawn, which illustrates the distribution of the data. As can be seen from Figure 4, the CCHMOPSO shows a significant improvement over the other four algorithms in the test problems ZDT1, ZDT2, ZDT4, ZDT6, UF1, UF2, UF5, UF7, UF9, and UF10. The lower the mean value of IGD and the shorter the box plot in the figure show that the IGD value obtained by the algorithm is better and has a more consistent result. In other test problems, except for DTLZ1, DTLZ2, DTLZ3, and DTLZ5, it is hard to see the difference between the effects of CCHMOPSO, NSGA-II, MOEAIGDNS, and SPEA2, while the performance of MOEAD is obviously poor. In general, CCHMOPSO gives better results than the other four algorithms.

As shown in Figure 5, convergence diagrams of five algorithms on test problems UF2, UF3, and ZDT6 are drawn. It is observed in the figure that CCHMOPSO converges faster than the other four algorithms because the combination method is used to select learning samples to effectively maintain the diversity of the population. At the same time, MOEAD has a faster convergence rate on the test problems UF3 and ZDT6, because the heuristic method adopted by the algorithm accelerates the convergence speed of the algorithm. The figure shows that each algorithm records the IGD value 10 times at a certain time interval between function evaluations. It can be seen that CCHMOPSO proposed in this study has a good convergence speed, which indicates that the three strategies proposed in CCHMOPSO can balance convergence and diversity well.

As can be seen from Figures 6 and 7, the Pareto peak surfaces of the CCHMOPSO, NSGA-II, MOEAIGDNS, SPEA2, and MOEAD algorithms are plotted in the dual-objective test problems ZDT2 and ZDT4. The true Pareto front of the test problem is drawn as a continuous straight line.  Figure 6 shows the true Pareto front for the test problem ZDT1, and only the CCHMOPSO proposed in this study almost completely fuses the true Pareto front, while the other four algorithms have almost no fusion for that true Pareto front. The distribution effect of CCHMOPSO is the best, mainly because it can well balance convergence and diversity. It can be observed from Figure 7 that the true Pareto front of ZDT2 is not completely covered by the other four MOEAs except CCHMOPSO, which almost completely covers the true Pareto front. From the above two figures, it is found that compared with the four other algorithms, only the approximate Pareto front of CCHMOPSO can be evenly distributed on the true Pareto front. The main reason is that they can improve the particle searchability using the combination method and maintaining the external archive strategy. In most test problems, because CCHMOPSO has good diversity and convergence, it can better approach the true Pareto front. It is noteworthy that CCHMOPSO obtains the best IGD value compared with the other four algorithms in both test problems, while it has the best overall performance.

### 4.4. Comparison with Four Multi-Objective Particle Swarm Optimization Algorithms

In the previous section, it was verified through experiments that CCHMOPSO performed better than these four MOEAs on most of the test problems of the DTLZ, UF, and ZDT series of test problems. However, the preceding experiments alone are not sufficient to demonstrate the advantages of CCHMOPSO. To further prove the advantages of CCHMOPSO, we compare it with four other MOPSOs. As shown in Tables 4 and 5, they give the mean and standard deviation of IGD values and HV values of the five algorithms in 22 test problems. Then, the best IGD and HV values of the five algorithms in 22 test problems are recorded, and the IGD and HV values of the corresponding algorithms are marked in bold.

It can be seen from Tables 4 and 5 that under 22 benchmark test problems, the overall performance of CCHMOPSO proposed in this article is better than the other four algorithms, namely CMOPSO, MOPSOCD, MPSOD, and NMPSO. As can be seen from the IGD values, CCHMOPSO, CMOPSO, and NMPSO achieve optimal IGD values on 12, 7, and 3 of the 22 test problems, respectively. For MOPSOCD and MPSOD, the results are not good on the DTLZ, UF, and ZDT series of test problems. The IGD values obtained by CCHMOPSO and CMOPSO are relatively better than the other three algorithms. For ZDT1-ZDT2 and ZDT6, the effect of CCHMOPSO is worse than CMOPSO, but better than other algorithms. For solving DTLZ6 PFs, CCHMOPSO performs best, because the central control strategy proposed by this algorithm can effectively search for the global optimum. One-to-one comparison shows that CCHMOPSO has better performance than CMOPSO, MOPSOCD, MPSOD, and NMPSO in 14, 16, 20, and 15 of the 22 comparisons. Meanwhile, CCHMOPSO is surpassed by CMOPSO, MOPSOCD, MPSOD, and NMPSO for 8, 6, 2, and 7 times, respectively. From the aspect of index IGD, it is proved that CCHMOPSO is better than the other four MOPSOs on most of the 22 test problems.

It can be seen from Table 5 that the comparison result of using index HV is similar to that of index IGD. As can be seen from the HV value, CMOPSO and NMPSO have the best performance in 4 and 5 times, respectively, while CCHMOPSO has 11 best performance. MOPSOCD and MPSOD perform worse than the other three algorithms on 22 test problems. In addition, in the test problems DTLZ1, DTLZ3, ZDT1, ZDT2, and ZDT6, CCHMOPSO is better for the measurement index IGD value, but slightly worse than the optimal algorithm. In test problem ZDT3, the IGD value of our CCHMOPSO is slightly worse, but it has the best overall performance. Therefore, CCHMOPSO is still superior to these four types of MOPSOs in solving these 22 test problems.

According to Figure 8, it can be seen that the CCHMOPSO proposed in this study has a significant improvement over the other four algorithms in the test problems ZDT4, UF1, UF2, UF5, UF7, UF8, UF9, and UF10. It is worth noting that the lower the IGD value and the shorter the box plot in the figure, it means that the algorithm has obtained a better average IGD value and at the same time has a more consistent result. In other test problems, except for the test problems DTLZ2 and DTLZ5, the effects of CCHMOPSO, CMOPSO, and NMPSO are better, while the performance of MOPSOCD and MPSOD is relatively poor. These figures further prove that CCHMOPSO's data results are better, and it also shows that it has better overall performance than other four algorithms on 22 test problems.

As shown in Figure 9, the convergence graphs of five algorithms on the test problems UF2, UF3, and ZDT6 are drawn. The figure shows that each algorithm records the IGD value 10 times at a certain time interval between function evaluations. It is observed from the figure that CCHMOPSO better balances the global search and local exploitation capabilities compared with the other four algorithms, resulting in better convergence of the algorithm. The CCHMOPSO proposed in this study has good convergence, mainly because the three strategies proposed in CCHMOPSO can balance convergence and diversity well.

As shown in Figures 10 and 11, the Pareto peak surfaces of CCHMOPSO, CMOPSO, MOPSOCD, MPSOD, and NMPSO are drawn in the dual-objective test problems ZDT2 and ZDT4. The true Pareto front of these test problems is plotted as a continuous straight line. It is observed from Figure 10 that the true Pareto front of ZDT2, except that CMOPSO and CCHMOPSO, can cover the true Pareto front very well, and the other three comparison algorithms have poor coverage of the true Pareto front. It can be seen intuitively from the figure that the approximate Pareto front of CCHMOPSO and CMOPSO is evenly distributed on the true Pareto front, mainly because they have the better convergence. It can be seen from Figure 11 that in ZDT4, except for CCHMOPSO, which can cover the true Pareto front, the other four comparison algorithms hardly approach the true Pareto front. Compared with the other four algorithms, this can intuitively show that CCHMOPSO has the best convergence effect, mainly because it uses the combination method to update the learning samples and improve the algorithm searchability. Due to incorrect convergence of CMOPSO, MOPSOCD, MPSOD, and NMPSO, their distributions do not perform well. It is worth noting that the overall performance of the CCHMOPSO proposed in this study is the best from the point of view of the metric IGD value and HV value. Therefore, CCHMOPSO obtains good convergence speed, and it can well balance convergence and diversity.

## 5. Conclusion

This study proposes a hybrid multi-objective particle swarm optimization with a central control strategy, which uses three strategies to improve the MOPSO. Firstly, the perturbation strategy is adopted to enable the particles in the population to obtain a wider search range, and at the same time, it can also prevent the population from trapping in the local optimum. Through the individual best particle update strategy of the combined method, the searchability of the algorithm is effectively improved, and the diversity of the population is also increased. Then, using the central control strategy to update the external archive, the archive can effectively store nondominated solutions. The experimental results on 22 test problems show that compared with the existing MOPSOs and classic MOEAs, CCHMOPSO has better overall performance.

## Figures and Tables

**Figure 1:** Pareto front of a set of solutions in a bi-objective space.

**Figure 2:** Deletion mechanism in the external archive.

**Figure 3:** CCHMOPSO's flowchart.

**Figure 4:** Box plot for the statistical results for IGD on 22 test problems.

**Figure 5:** Convergence graph for UF2, UF3 and ZDT6.

**Figure 6:** On the dual-target ZDT1, the true Pareto front is shown as a continuous straight line, and Pareto fronts are generated by (a) MOEAIGDNS, (b) SPEA2, (c) NSGA-II, (d) MOEAD, and (e) CCHMOPSO on ZDT1.

**Figure 7:** On the dual-target ZDT2, the true Pareto front is shown as a continuous straight line, and Pareto fronts are generated by (a) MOEAIGDNS, (b) SPEA2, (c) NSGA-II, (d) MOEAD, and (e) CCHMOPSO on ZDT2.

**Figure 8:** Box plot for the statistical results for IGD on 22 test problems.

**Figure 9:** Convergence graph for UF2, UF3, and ZDT6.

**Figure 10:** On the dual-target ZDT2, the true Pareto front is shown as a continuous straight line, and Pareto fronts are generated by (a) CMOPSO, (b) MOPSOCD, (c) MPSOD, (d) NMPSO, and (e) CCHMOPSO on ZDT2.

**Figure 11:** On the dual-target ZDT4, the true Pareto front is shown as a continuous straight line, and Pareto fronts are generated by (a) CMOPSO, (b) MOPSOCD, (c) MPSOD, (d) NMPSO, and (e) CCHMOPSO on ZDT4.

**Table 1:** Parameter settings for all the algorithms.

Algorithms	Parameter settings
MOEAIGDNS	*η*_*c*_=*η*_*m*_=20, *p*_*c*_=1.0, *p*_*m*_=(1/*n*)
SPEA2	*η*_*c*_=*η*_*m*_=20, *p*_*c*_=1.0, *p*_*m*_=1.0, *p*=0.5
NSGA-II	*η*_*c*_=*η*_*m*_=20, *p*_*c*_=0.9, *p*_*m*_=(1/*n*)
MOEAD	*η*_*m*_=20, *p*_*m*_=(1/*n*), *T*=20, *F*=0.5
CMOPSO	*w*=0.4, *R*_1_, *R*_2_ ∈ [0,1]
MOPSOCD	*R*_1_, *R*_2_ ∈ [0,1]
MPSOD	*η*_*m*_=20, *p*_*m*_=0.1, *c*_1_=*c*_2_=2.0, *w* ∈ [0.1, 0.9]
NMPSO	*η*_*m*_=20, *p*_*m*_=(1/*n*), *c*_1_, *c*_2_, *c*_3_ ∈ [1.5, 2.5], *w* ∈ [0.1, 0.5]
CCHMOPSO	*w*=0.4, *c*_1_=*c*_2_=2.0, div=50

**Table 2:** On test problems ZDT, DTLZ, and UF, the mean and variance of IGD measures obtained by CCHMOPSO and four MOEAs running for 30 times are presented in this study.

Problem	*N*	*M*	*D*	MOEAIGDNS	SPEA2	NSGA-II	MOEAD	CCHMOPSO
DTLZ1	200	3	7	9.2547*e* − 1 (3.91*e* − 1)	**3.1660*e*** − **1 (2.53*e*** − **1)**	3.3201*e* − 1 (2.09*e* − 1)	3.4069e − 1 (4.71e − 1)	7.3666e + 0 (1.93e + 0)
DTLZ2	200	3	12	4.3409*e* − 2 (1.22*e* − 3)	4.0048*e* − 2 (6.08*e* − 4)	5.0728*e* − 2 (1.21*e* − 3)	**3.9605e** − **2 (7.92e** − **4)**	1.8109 e − 1 (1.50e − 2)
DTLZ3	200	3	12	2.8805*e* + 1 (7.97*e* + 0)	1.7268*e* + 1 (4.89*e* + 0)	**1.4015*e*** **+** **1 (4.63*e*** **+** **0)**	1.8939e + 1 (1.19e + 1)	1.3511e + 2 (8.87e + 0)
DTLZ4	200	3	12	**4.3770*e*** − **2 (1.05*e*** − **3)**	1.0735*e* − 1 (1.73*e* − 1)	4.9686*e* − 2 (1.39*e* − 3)	4.0063e − 1 (2.79e − 1)	2.2261e − 1 (2.40e − 2)
DTLZ5	200	3	12	5.7369*e* − 3 (7.50*e* − 4)	4.5843*e* − 3 (5.23*e* − 4)	**3.9909*e*** − **3 (3.78*e*** − **4)**	2.0192e − 2 (8.37e − 4)	4.8917e − 2 (1.26e − 2)
DTLZ6	200	3	12	5.4930*e* − 2 (1.14*e* − 1)	3.4740*e* − 2 (1.46*e* − 1)	**4.1062*e*** − **3 (2.08*e*** − **3)**	4.8427e − 2 (1.52e − 1)	1.1330e − 2 (2.51e − 3)
DTLZ7	200	3	22	1.6234*e* − 1 (4.07*e* − 2)	**9.1755*e*** − **2 (1.71*e*** − **2)**	1.1432*e* − 1 (1.95*e* − 2)	1.9843e − 1 (2.11e − 1)	1.3414e − 1 (1.66e − 2)
UF1	200	2	30	1.1728*e* − 1 (2.75*e* − 2)	1.1571*e* − 1 (2.57*e* − 2)	1.1182*e* − 1 (1.87*e* − 2)	3.4835e − 1 (1.14e − 1)	**3.0912e** − **2 (1.02e** − **2)**
UF2	200	2	30	7.6132*e* − 2 (5.06*e* − 3)	6.9040*e* − 2 (5.24*e* − 3)	6.5446*e* − 2 (4.96*e* − 3)	2.0211e − 1 (7.53e − 2)	**2.4220e** − **2 (3.87e** − **3)**
UF3	200	2	30	4.6565*e* − 1 (1.35*e* − 2)	4.3997*e* − 1 (2.02*e* − 2)	4.4100*e* − 1 (2.24*e* − 2)	3.3700e − 1 (2.52e − 2)	**9.8163e** − **2 (2.85e** − **2)**
UF4	200	2	30	8.8403*e* − 2 (2.82*e* − 3)	8.0429*e* − 2 (2.41*e* − 3)	8.1366*e* − 2 (3.07*e* − 3)	1.1689e − 1 (4.85e − 3)	**6.3123e** − **2 (4.66e** − **3)**
UF5	200	2	30	1.2218*e* + 0 (3.45*e* − 1)	9.0832*e* − 1 (2.55*e* − 1)	8.4678*e* − 1 (2.68*e* − 1)	1.4132e + 0 (2.60e − 1)	**3.4936e** − **1 (1.31e** − **1)**
UF6	200	2	30	6.3514*e* − 1 (1.23*e* − 1)	5.7381*e* − 1 (1.00*e* − 1)	5.3083*e* − 1 (9.32*e* − 2)	6.0455e − 1 (2.12e − 1)	**2.5443e** − **1 (9.86e** − **2)**
UF7	200	2	30	1.7392*e* − 1 (8.52*e* − 2)	1.3931*e* − 1 (7.37*e* − 2)	1.5873*e* − 1 (8.56*e* − 2)	4.8541e − 1 (1.11e − 1)	**3.3066e** − **2 (6.76e** − **3)**
UF8	200	3	30	3.8403*e* − 1 (4.31*e* − 2)	3.1338*e* − 1 (4.21*e* − 2)	**3.0619*e*** − **1 (3.74*e*** − **2)**	5.8169e − 1 (2.69e − 1)	3.1127e − 1 (3.25e − 2)
UF9	200	3	30	5.0578*e* − 1 (4.50*e* − 2)	4.5228*e* − 1 (5.61*e* − 2)	4.3576*e* − 1 (7.37*e* − 2)	5.1904e − 1 (9.16e − 2)	**2.2239e** − **1 (4.11e** − **2)**
UF10	200	3	30	1.7872*e* + 0 (4.30*e* − 1)	1.4254*e* + 0 (4.56*e* − 1)	1.2798*e* + 0 (3.66*e* − 1)	7.4165e − 1 (7.37e − 2)	**7.2137e** − **1 (1.69e** − **2)**
ZDT1	200	2	30	7.3411*e* − 2 (1.34*e* − 2)	4.0594*e* − 2 (6.48*e* − 3)	3.5803*e* − 2 (5.87*e* − 3)	1.8466e − 1 (6.82e − 2)	**4.9539e** − **3 (4.40e** − **4)**
ZDT2	200	2	30	1.5227*e* − 1 (2.75*e* − 2)	8.2136*e* − 2 (4.38*e* − 2)	7.0364*e* − 2 (2.05*e* − 2)	5.6916e − 1 (6.67e − 2)	**5.2140e** − **3 (6.11e** − **4)**
ZDT3	200	2	30	6.7653*e* − 2 (1.30*e* − 2)	3.8623*e* − 2 (8.63*e* − 3)	**3.2682*e*** − **2 (8.98*e*** − **3)**	1.6165e − 1 (4.93e − 2)	2.0293e − 1 (5.07e − 3)
ZDT4	200	2	10	2.1178*e* + 0 (7.84*e* − 1)	8.7986*e* − 1 (3.71*e* − 1)	1.0316*e* + 0 (4.46*e* − 1)	5.4565e − 1 (1.74e − 1)	**4.8758e** − **3 (3.54e** − **4)**
ZDT6	200	2	10	1.2284*e* + 0 (2.36*e* − 1)	5.8271*e* − 1 (1.43*e* − 1)	5.1824*e* − 1 (1.56*e* − 1)	8.8109e − 2 (2.21e − 2)	**2.0407e** − **3 (2.73e** − **4)**
Best/all				1/22	2/22	5/22	1/22	13/22

**Table 3:** On test problems ZDT, DTLZ, and UF, the mean and variance of HV measures obtained by CCHMOPSO and four MOEAs running for 30 times are presented in this study.

Problem	*N*	M	D	MOEAIGDNS	SPEA2	NSGA-II	MOEAD	CCHMOPSO
DTLZ1	200	3	7	1.5390e − 2 (4.71e − 2)	3.0780e − 1 (3.16e − 1)	2.4332e − 1 (2.81e − 1)	**4.1676e** − **1 (3.48e** − **1)**	0.0000e + 0(0.00e + 0)
DTLZ2	200	3	12	5.5680e − 1 (2.17e − 3)	**5.6266e** − **1 (1.46e** − **3)**	5.4486e − 1 (2.67e − 3)	5.6136e − 1 (2.17e − 3)	3.3442e − 1 (2.18e − 2)
DTLZ3	200	3	12	0.0000e + 0 (0.00e + 0)	0.0000e + 0 (0.00e + 0)	0.0000e + 0 (0.00e + 0)	0.0000e + 0 (0.00e + 0)	0.0000e + 0 (0.00e + 0)
DTLZ4	200	3	12	**5.5889e** − **1 (2.36e** − **3)**	5.3296e − 1 (7.41e − 2)	5.4724e − 1 (3.26e − 3)	4.0280e − 1 (1.34e − 1)	4.1743e − 1 (2.41e − 3)
DTLZ5	200	3	12	1.9767e − 1 (5.08e − 4)	1.9866e − 1 (5.34e − 4)	**1.9955e** − **1 (3.28e** − **4)**	1.8844e − 1 (1.05e − 3)	1.3584e − 1 (1.81e − 2)
DTLZ6	200	3	12	1.7100e − 1 (3.51e − 2)	1.8934e − 1 (3.64e − 2)	**1.9968e** − **1 (2.18e** − **3)**	1.7738e − 1 (3.44e − 2)	1.9010e − 1 (5.31e − 3)
DTLZ7	200	3	22	2.1400e − 1 (1.50e − 2)	2.4357e − 1 (9.19e − 3)	2.3141e − 1 (9.04e − 3)	2.2103e − 1 (2.10e − 2)	**2.5112e** − **1 (6.01e** − **3)**
UF1	200	2	30	5.4335e − 1 (3.83e − 2)	5.5028e − 1 (3.60e − 2)	5.6453e − 1 (2.84e − 2)	3.9709e − 1 (6.45e − 2)	**6.8094e** − **1 (1.55e** − **2)**
UF2	200	2	30	6.2596e − 1 (5.91e − 3)	6.3649e − 1 (5.08e − 3)	6.3995e − 1 (5.08e − 3)	5.6569e − 1 (3.08e − 2)	**6.8316e** − **1 (8.18e** − **3)**
UF3	200	2	30	1.9441e − 1 (1.04e − 2)	2.1660e − 1 (1.36e − 2)	2.1166e − 1 (1.94e − 2)	2.9743e − 1 (3.39e − 2)	**6.0783e** − **1 (3.31e** − **2)**
UF4	200	2	30	3.2380e − 1 (3.54e − 3)	3.3426e − 1 (3.08e − 3)	3.3338e − 1 (3.57e − 3)	2.8211e − 1 (6.22e − 3)	**3.6066e** − **1 (6.77e** − **3)**
UF5	200	2	30	2.4567e − 3 (1.22e − 2)	6.5804e − 3 (1.72e − 2)	2.3117e − 2 (4.58e − 2)	0.0000e + 0 (0.00e + 0)	**1.4021e** − **1 (9.22e** − **2)**
UF6	200	2	30	1.7631e − 2 (1.90e − 2)	3.2667e − 2 (2.91e − 2)	4.1639e − 2 (3.29e − 2)	6.8170e − 2 (6.77e − 2)	**2.0239e** − **1 (6.65e** − **2)**
UF7	200	2	30	3.7237e − 1 (7.28e − 2)	4.0160e − 1 (6.58e − 2)	3.9115e − 1 (7.15e − 2)	2.1124e − 1 (5.54e − 2)	**5.3892e** − **1 (9.31e** − **3)**
UF8	200	3	30	2.5396e − 1 (3.49e − 2)	2.6879e − 1 (5.13e − 2)	**2.7227e** − **1 (4.12e** − **2)**	1.5694e − 1 (6.81e − 2)	2.5969e − 1 (2.24e − 2)
UF9	200	3	30	2.6132e − 1 (2.97e − 2)	2.9819e − 1 (4.32e − 2)	3.1274e − 1 (6.12e − 2)	2.8664e − 1 (5.52e − 2)	**5.0003e** − **1 (3.58e** − **2)**
UF10	200	3	30	0.0000e + 0 (0.00e + 0)	0.0000e + 0 (0.00e + 0)	1.5891e − 6 (8.70e − 6)	3.3147e − 2 (2.36e − 2)	**9.2144e** − **2 (2.68e** − **3)**
ZDT1	200	2	30	6.2402e − 1 (1.72e − 2)	6.6851e − 1 (8.70e − 3)	6.7472e − 1 (7.96e − 3)	5.3338e − 1 (5.84e − 2)	**7.1843e** − **1 (6.81e** − **4)**
ZDT2	200	2	30	2.5471e − 1 (2.56e − 2)	3.3647e − 1 (3.90e − 2)	3.4900e − 1 (2.70e − 2)	9.3271e − 2 (2.18e − 2)	**4.4170e** − **1 (1.55e** − **3)**
ZDT3	200	2	30	5.5577e − 1 (9.21e − 3)	5.7319e − 1 (4.99e − 3)	5.8430e − 1 (2.41e − 2)	5.6123e − 1 (5.67e − 2)	**6.5549e** − **1 (2.44e** − **3)**
ZDT4	200	2	10	0.0000e + 0 (0.00e + 0)	5.2117e − 2 (6.86e − 2)	3.9236e − 2 (7.70e − 2)	1.7020e − 1 (1.23e − 1)	**7.1881e** − **1 (5.42e** − **4)**
ZDT6	200	2	10	7.3169e − 4 (4.01e − 3)	1.8248e − 2 (2.58e − 2)	3.2482e − 2 (3.70e − 2)	2.7381e − 1 (2.41e − 2)	**3.8527e** − **1 (1.12e** − **3)**
Best/all				1/22	1/22	3/22	1/22	15/22

**Table 4:** On the test problems ZDT, DTLZ, and UF, the mean and variance of IGD measures obtained by CCHMOPSO and four MOPSOs running for 30 times.

Problem	*N*	*M*	*D*	CMOPSO	MOPSOCD	MPSOD	NMPSO	CCHMOPSO
DTLZ1	200	3	7	1.6354e + 1 (4.40e + 0)	1.8583e + 1 (3.91e + 0)	1.0384e + 1 (2.29e + 0)	**5.8743e** **+** **0 (3.34e** **+** **0)**	7.3666e + 0 (1.93e + 0)
DTLZ2	200	3	12	**4.1471e** − **2 (5.50e** − **4)**	9.2976e − 2 (1.12e − 2)	4.5744e − 2 (1.82e − 3)	5.5638e − 2 (2.03e − 3)	1.8109e − 1 (1.50e − 2)
DTLZ3	200	3	12	1.9270e + 2 (3.38e + 1)	1.2913e + 2 (3.96e + 1)	1.4835e + 2 (1.32e + 1)	**1.1520e** **+** **2 (1.88e** **+** **1)**	1.3511e + 2 (8.87e + 0)
DTLZ4	200	3	12	**4.3528e** − **2 (1.56e** − **3)**	3.1908e − 1 (4.46e − 2)	1.2958e − 1 (3.07e − 2)	5.7773e − 2 (2.12e − 3)	2.2261e − 1 (2.40e − 2)
DTLZ5	200	3	12	**4.5711e** − **3 (2.32e** − **4)**	3.7335e − 2 (9.98e − 3)	5.5848e − 2 (6.48e − 3)	6.8616e − 3 (1.06e − 3)	4.8917e − 2 (1.26e − 2)
DTLZ6	200	3	12	2.3831e − 1 (3.97e − 1)	1.9092e − 1 (3.40e − 1)	1.1505e + 0 (3.80e − 1)	1.2699e − 2 (2.27e − 3)	**1.1330e** − **2 (2.51e** − **3)**
DTLZ7	200	3	22	4.9477e − 2 (3.35e − 3)	9.7770e − 2 (9.05e − 2)	5.6014e − 1 (1.50e − 1)	**4.6016e** − **2 (2.12e** − **3)**	1.3414e − 1 (1.66e − 2)
UF1	200	2	30	1.0688e − 1 (3.00e − 2)	6.4317e − 1 (1.21e − 1)	2.7257e − 1 (4.65e − 2)	1.2485e − 1 (1.37e − 2)	**3.0912e** − **2 (1.02e** − **2)**
UF2	200	2	30	6.1861e − 2 (7.31e − 3)	1.3780e − 1 (1.37e − 2)	1.1285e − 1 (1.08e − 2)	8.5789e − 2 (6.14e − 3)	**2.4220e** − **2 (3.87e** − **3)**
UF3	200	2	30	4.0343e − 1 (3.35e − 2)	3.6746e − 1 (5.74e − 2)	4.9750e − 1 (1.61e − 2)	3.4911e − 1 (4.64e − 2)	**9.8163e** − **2 (2.85e** − **2)**
UF4	200	2	30	1.1336e − 1 (9.80e − 3)	7.9528e − 2 (8.68e − 3)	9.9476e − 2 (4.79e − 3)	6.4582e − 2 (9.86e − 3)	**6.3123e** − **2 (4.66e** − **3)**
UF5	200	2	30	8.9886e − 1 (2.40e − 1)	3.9973e + 0 (2.96e − 1)	2.8538e + 0 (2.50e − 1)	1.5029e + 0 (5.35e − 1)	**3.4936e** − **1 (1.31e** − **1)**
UF6	200	2	30	3.7821e − 1 (5.36e − 2)	3.1206e + 0 (7.84e − 1)	1.3180e + 0 (2.28e − 1)	6.4338e − 1 (1.29e − 1)	**2.5443e** − **1 (9.86e** − **2)**
UF7	200	2	30	1.1138e − 1 (9.20e − 2)	6.3678e − 1 (1.29e − 1)	2.3429e − 1 (7.16e − 2)	2.3483e − 1 (1.96e − 1)	**3.3066e** − **2 (6.76e** − **3)**
UF8	200	3	30	5.7919e − 1 (7.51e − 2)	7.6172e − 1 (1.72e − 1)	5.5574e − 1 (4.34e − 2)	4.6532e − 1 (1.00e − 1)	**3.1127e** − **1 (3.25e** − **2)**
UF9	200	3	30	8.7747e − 1 (1.32e − 1)	8.3358e − 1 (1.09e − 1)	6.6695e − 1 (3.82e − 2)	4.6821e − 1 (6.41e − 2)	**2.2239e** − **1 (4.11e** − **2)**
UF10	200	3	30	4.3313e + 0 (4.79e − 1)	5.1104e + 0 (9.25e − 1)	4.0571e + 0 (4.13e − 1)	1.5475e + 0 (3.16e − 1)	**7.2137e** − **1 (1.69e** − **2)**
ZDT1	200	2	30	**2.9555e** − **3 (4.20e** − **4)**	7.8407e − 3 (2.82e − 2)	1.0216e − 1 (4.56e − 2)	3.1064e − 2 (1.11e − 2)	4.9539e − 3 (4.40e − 4)
ZDT2	200	2	30	**2.8456e** − **3 (2.73e** − **4)**	1.0420e − 1 (1.44e − 1)	1.2123e − 1 (6.68e − 2)	1.8649e − 2 (3.69e − 3)	5.2140e − 3 (6.11e − 4)
ZDT3	200	2	30	**3.9451e** − **3 (9.65e** − **4)**	3.9143e − 2 (5.68e − 2)	2.0405e − 1 (5.16e − 2)	9.2609e − 2 (2.25e − 2)	2.0293e − 1 (5.07e − 3)
ZDT4	200	2	10	2.0059e + 1 (6.48e + 0)	1.9360e + 1 (8.29e + 0)	3.8323e + 1 (7.06e + 0)	1.7546e + 1 (9.68e + 0)	**4.8758e** − **3 (3.54e** − **4)**
ZDT6	200	2	10	**1.5805e** − **3 (3.15e** − **5)**	3.8328e − 3 (3.08e − 3)	2.0893e − 2 (1.65e − 2)	2.2388e − 3 (1.71e − 4)	2.0407e − 3 (2.73e − 4)
Best/all				7/22	0/22	0/22	3/22	12/22

**Table 5:** On the test problems ZDT, DTLZ, and UF, the mean and variance of HV measures obtained by CCHMOPSO and four MOPSOs running for 30 times.

Problem	N	M	D	CMOPSO	MOPSOCD	MPSOD	NMPSO	CCHMOPSO
DTLZ1	200	3	7	0.0000e + 0 (0.00e + 0)	0.0000e + 0 (0.00e + 0)	0.0000e + 0 (0.00e + 0)	0.0000e + 0 (0.00e + 0)	0.0000e + 0 (0.00e + 0)
DTLZ2	200	3	12	5.5873e − 1 (1.38e − 3)	4.7940e − 1 (1.92e − 2)	5.4913e − 1 (3.77e − 3)	**5.6970e** − **1 (9.34e** − **4)**	3.3442e − 1 (2.18e − 2)
DTLZ3	200	3	12	0.0000e + 0 (0.00e + 0)	0.0000e + 0 (0.00e + 0)	0.0000e + 0 (0.00e + 0)	0.0000e + 0 (0.00e + 0)	0.0000e + 0 (0.00e + 0)
DTLZ4	200	3	12	5.5542e − 1 (3.36e − 3)	2.8437e − 1 (5.32e − 2)	4.3677e − 1 (3.62e − 2)	**5.6836e** − **1 (1.27e** − **3)**	4.1743e − 1 (2.41e − 3)
DTLZ5	200	3	12	**1.9894e** − **1 (2.30e** − **4)**	1.7022e − 1 (9.63e − 3)	1.4053e − 1 (9.30e − 3)	1.9812e − 1 (8.22e − 4)	1.3584e − 1 (1.81e − 2)
DTLZ6	200	3	12	1.4602e − 1 (8.74e − 2)	1.5957e − 1 (7.01e − 2)	6.9866e − 3 (2.63e − 2)	**1.9799e** − **1 (6.55e** − **4)**	1.9010e − 1 (5.31e − 3)
DTLZ7	200	3	22	2.7294e − 1 (2.73e − 3)	2.5967e − 1 (3.35e − 2)	6.4616e − 2 (3.89e − 2)	**2.8167e** − **1 (5.91e** − **4)**	2.5112e − 1 (6.01e − 3)
UF1	200	2	30	5.7327e − 1 (2.13e − 2)	7.3114e − 2 (6.50e − 2)	3.5345e − 1 (5.13e − 2)	5.3056e − 1 (2.43e − 2)	**6.8094e** − **1 (1.55e** − **2)**
UF2	200	2	30	6.4384e − 1 (8.88e − 3)	5.4501e − 1 (1.82e − 2)	5.8040e − 1 (1.21e − 2)	6.1737e − 1 (6.14e − 3)	**6.8316e** − **1 (8.18e** − **3)**
UF3	200	2	30	2.5742e − 1 (2.53e − 2)	2.6453e − 1 (4.42e − 2)	1.7555e − 1 (1.63e − 2)	2.8952e − 1 (3.95e − 2)	**6.0783e** − **1 (3.31e** − **2)**
UF4	200	2	30	2.8804e − 1 (1.27e − 2)	3.3192e − 1 (1.17e − 2)	3.0742e − 1 (5.54e − 3)	3.5766e − 1 (1.37e − 2)	**3.6066e** − **1 (6.77e** − **3)**
UF5	200	2	30	1.1860e − 2 (2.97e − 2)	0.0000e + 0 (0.00e + 0)	0.0000e + 0 (0.00e + 0)	0.0000e + 0 (0.00e + 0)	**1.4021e** − **1 (9.22e** − **2)**
UF6	200	2	30	1.5459e − 1 (6.45e − 2)	0.0000e + 0 (0.00e + 0)	0.0000e + 0 (0.00e + 0)	2.4309e − 2 (3.04e − 2)	**2.0239e** − **1 (6.65e** − **2)**
UF7	200	2	30	4.5152e − 1 (7.30e − 2)	2.7305e − 2 (3.84e − 2)	2.7968e − 1 (6.52e − 2)	3.4621e − 1 (1.31e − 1)	**5.3892e** − **1 (9.31e** − **3)**
UF8	200	3	30	1.6756e − 2 (2.12e − 2)	1.0655e − 2 (1.85e − 2)	5.0793e − 2 (1.96e − 2)	**2.7450e** − **1 (5.92e** − **2)**	2.5969e − 1 (2.24e − 2)
UF9	200	3	30	2.4592e − 2 (3.17e − 2)	3.7103e − 2 (3.62e − 2)	1.0811e − 1 (2.71e − 2)	3.0726e − 1 (6.30e − 2)	**5.0003e** − **1 (3.58e** − **2)**
UF10	200	3	30	0.0000e + 0 (0.00e + 0)	0.0000e + 0 (0.00e + 0)	0.0000e + 0 (0.00e + 0)	0.0000e + 0 (0.00e + 0)	**9.2144e** − **2 (2.68e** − **3)**
ZDT1	200	2	30	**7.2023e** − **1 (6.89e** − **4)**	7.1485e − 1 (3.46e − 2)	5.7486e − 1 (6.04e − 2)	6.8834e − 1 (1.28e − 2)	7.1843e − 1 (6.81e − 4)
ZDT2	200	2	30	**4.4481e** − **1 (4.64e** − **4)**	3.4118e − 1 (1.42e − 1)	2.9361e − 1 (7.47e − 2)	4.3608e − 1 (2.36e − 3)	4.4170e − 1 (1.55e − 3)
ZDT3	200	2	30	5.9983e − 1 (1.34e − 3)	5.7793e − 1 (4.10e − 2)	4.4817e − 1 (4.74e − 2)	5.7050e − 1 (8.22e − 3)	**6.5549e** − **1 (2.44e** − **3)**
ZDT4	200	2	10	0.0000e + 0 (0.00e + 0)	0.0000e + 0 (0.00e + 0)	0.0000e + 0 (0.00e + 0)	0.0000e + 0 (0.00e + 0)	**7.1881e** − **1 (5.42e** − **4)**
ZDT6	200	2	10	**3.9034e** − **1 (3.50e** − **5)**	3.8822e − 1 (2.92e − 3)	3.7169e − 1 (1.57e − 2)	3.8981e − 1 (1.46e − 4)	3.8527e − 1 (1.12e − 3)
Best/all				4/22	0/22	0/22	5/22	11/22

## Data Availability

No data were used to support this study.
